The article "Nursing Research of Optic Canal Decompression Operation under Nasal Endoscopic Medical Treatment Based on Intelligent Internet of Things for Traumatic Vision Disorders" was retracted in 2023. Reasons: signs of a paper mill; suspected computer-generated content; unreliable results or conclusions; lack of ethics approval or compliance.

# Nursing Research of Optic Canal Decompression Operation under Nasal Endoscopic Medical Treatment Based on Intelligent Internet of Things for Traumatic Vision Disorders

**DOI:** 10.1155/2021/9999863

**Published:** 2021-07-01

**Authors:** Yu Liu, Yanchun Zhao, Xia Gong, Ying Zhang

**Affiliations:** ^1^Department of Neurology, Jinan Third People's Hospital, Jinan 250101, Shandong, China; ^2^Department of Public Health, Jinan Hospital of Traditional Chinese Medicine, Jinan 250012, Shandong, China; ^3^Department of Gynecology and Social Security, Qingdao Jimo District Level 7 Health Center, Qingdao 266011, Shandong, China; ^4^Ophthalmology Department of Jinan Second People's Hospital, Jinan 250001, Shandong, China

## Abstract

Traumatic vision is an important factor that causes people to have a vision. In our country, the vast majority of vision is caused by trauma. To understand the role of optic nerve decompression in the treatment of traumatic visual disturbances based on the pathological states of traumatic visual disturbances and intelligent Internet of tumors medical nasal endoscopy optic nerve decompression. This article collects relevant information by investigating patients, investigating relevant literature, interviewing professionals, etc., constructing a case template and using a comprehensive quantitative and qualitative analysis method to create a damage assessment matrix. The results of the study found that most traumatic vision disorders occur in the young and middle-aged stage, which is more than three times that of other age groups. The permanent blindness rate of patients reaches 8%, which is extremely harmful. Optic canal decompression surgery can play a great role in the treatment of patients. It can greatly reduce the patient's neurological damage. The effect is about 30% higher than that of general treatment methods, and it can also play a certain role in the prognosis of rehabilitation. It can effectively prevent related postoperative complications. This shows that optic canal decompression in the treatment of traumatic vision disorders should attract people's attention and increase research and development efforts and promotion efforts so that optic canal decompression can be used in the diagnosis and treatment of patients with traumatic vision disorders based on smart Internet of things China can play a greater role.

## 1. Introduction

Cognitive function is an important prerequisite for people to perceive the peripheral world and to adapt to the objective environment. A specific injury factor, such as a head injury and stroke, causes damage to the brain tissue, often causing cognitive dysfunction in the patient, resulting in difficulty in perceiving the patient and adapting to the external environment. Life and society can live independently, work hard, and even constitute obstacles [1, 2]. Various cognitive dysfunctions appear in the human head after trauma, such as emotional disturbance, memory loss, and decreased concentration. There are many factors that affect intellectual impairment. Brain stem damage and intracranial hematoma have a significant impact on mental disability, causing vision problems and possibly affecting human life, health, and safety. People need to pay attention [3].

With the development of science and technology, especially the application of imaging technology in the medical field, it provides a reliable guarantee for doctors at the risk of optic canal decompression surgery [4]. In order to reduce the risk of optic nerve decompression surgery based on previous nasal endoscopic surgery, virtual endoscopes based on CT images enter the lumen of the sphenoid sinus before surgery and observe the canine and internal carotid arteries of the optic canal. The adjacent relationship between the base, the pituitary gland, etc., predicts the level of risk of surgery and plans the approach to surgery. And input CT images and virtual endoscopy images into the navigation equipment, trying to study the role of virtual endoscopy technology and navigation technology in reducing the risk of surgery, planning the surgical approach, and reducing surgical trauma [5].

Regarding the impact of traumatic visual impairment on patients, experts at home and abroad also have many studies: Cheng and Jia believe that traumatic visual impairment causes extremely serious damage to people. After treatment, more care should be given to patients. Patients admitted to a hospital in northern Anhui received relevant psychological care for one year to study whether they had a positive effect on the prognosis of traumatic visual impairment. The results showed that after psychological care, the patient's neurological deficit score increased significantly, indicating that psychological care is effective. Traumatic visual impairment can play a role in promoting the recovery of patients' neurological function and daily living ability [6]; Li et al. investigated the role of Shuxuening injection in patients with traumatic vision, selecting 30 cases of traumatic vision. Patients with disabilities were divided into experimental and observational groups. When the patients were treated, the experimental group was injected with Shuxuening injection, the observation group did not inject, and the two groups of patients recorded various physical functions after treatment. The experimental results found that the neurological deficits of patients injected with Shuxuening injection were lower than those of the observation group, and they believed that Shuxuening injection could play a positive role in patients with traumatic visual impairment [7]; Tu and Su made statistics on patients with traumatic visual impairment. According to the patient's gender, age, morbidity, and recurrence rate, it classified the patients and found that the incidence of traumatic visual impairment is about 0.58%–0.61%, which shows that traumatic visual impairment poses a threat to people's health [8]. These studies have a certain reference basis for this article, but due to insufficient samples of these studies, too much emphasis on theories, and unreasonable practical programs, there are too many variables in the study, and the conclusions are unconvincing.

This article is primarily to study the impact of optical nerve decompression surgery visualization on the treatment of traumatic vision through the visualization of medically assisted Internet surgical design, reducing the risk of surgery. Combining medicine, biology, computing, instrumentation, and mechanics related disciplines, relying on computer graphics and image technology, segmentation and reconstruction technology, virtual roaming technology, etc., display the patient's information according to the doctor's requirements, and help the doctor to plan the operation. Provide great help to doctors in surgery, reduce the risk to patients, reduce unnecessary pain for patients, and increase the success rate of surgery.

## 2. Nursing Methods of Optic Canal Decompression for Traumatic Vision Disorders

### 2.1. IoT Medical Nasal Endoscopy

Visual acuity is a more accurate function of form perception. It can be divided into central visual acuity and peripheral visual acuity. Central visual acuity is obtained through the center of the macula. Peripheral visual acuity refers to the functions of the retina other than the macula. Therefore, vision is one of the specific manifestations of visual function. The visual impairment, although very slight, also shows that the visual function is affected.

Mono's Internet uses information recognition techniques such as sensors and runs through a wireless network between patients and medical staff, medical institutions, and medical devices. Through the comprehensive application of handwriting recognition, identity recognition, sensor wireless network, and other Internet of Things technologies, identification, local positioning, monitoring, and management of special populations in hospitals, medical equipment, medical waste, and medicines have been carried out. You can play the following aspects in this process: diagnostic and treatment entry points, patient ID line bar codes, mobile doctor orders, mobile test sample management, mobile drug management, infant theft prevention, medical records, data dialing and storage, nursing program management, and so on [9]. It can monitor various human conditions in the medical field and transmit data to different terminals. Its main application is to monitor the human body and measure normal parameters. The monitored items include not only patients, but also healthy people [10].

As shown in Figure 1, endoscopes can be divided into different types according to function, reach, and structure. According to different functions, it can be divided into observation mirror and work mirror and the work mirror can be used to treat cerebral hemorrhage. In addition to the observation mirror function, there are working channels in the working mirror. Through working channels, you can complete various functions such as surgery, flushing, aspiration, and stasis [11]. According to the different viewing angles of the endoscope, it is divided into 0°, 30°, 45°, 70°, 120° endoscope. Neuroendoscopy is mainly composed of lens body, light source, imaging system, and image recording device.

1. Scope: the scope of neuroendoscopy includes rigid endoscope, flexible endoscope, and observation peeling mirror [12]. Rigid endoscopes are used to treat cerebral hemorrhage. Rigid endoscopes use multiple cylindrical lens systems to image. The outer diameter is generally 2∼8 mm. It can complete the functions of illumination, washing, suction, working channel, etc., and its length is generally 130∼300 mm. The endoscopic surgical instrument enters the operating field along the inside and outside of the endoscope, and the operation is completed under the supervision of the monitor. We usually use 0° and 30 degrees lenses for observation and surgery.
2. Light source: the brightness of the light directly affects the quality of the image, from the first endoscope using candle light to the later invention of the light bulb and the use of incandescent bulbs, and then to the widespread use of metal halide lamps and ultrahigh voltage short-arc lamps in the 1960s. For applications, neuroendoscopy lighting systems are constantly evolving [13].
3. Imaging system: the imaging system includes a camera, a camera system, and a display. The camera is connected to the eyepiece of the neuroendoscope, and the image is transmitted to the display through the camera system host; the display shows that the image collected by the camera is the “eye” of the surgeon, and it is mostly placed directly in front of the surgeon's operating position. The distance should not exceed 2 meters to facilitate observation [14].
4. Storage system: image recording device and computer management system. The image recording apparatus can be used to record and store full information, including video devices, optical discs, hard disk storage media and printing devices and can be used to convert an operating image to a digital signal or directly print to a photo to store, display, or expose data [15]. Some camera system hosts integrate the function of an image recording device, and directly output images or videos to U disk and hard disk, which is convenient to use.

Aiming at the problem that the Snake algorithm will not converge when the initial position is not appropriate, and the search range is limited, this paper uses the GVF model to make up for the above shortcomings. This model uses the gradient vector on the image to diffuse outward to increase the capture area, a recessed area that is deep in the contour of the target. Therefore, the GVF field can expand the range of target detection.

Set *f*(*x*, *y*) as the edge-mapped image of the image *I*(*x*, *y*), the *f*(*x*, *y*) general value here is |∇(*Gσ*(*x*, *y*)*∗I*(*x*, *y*))|^2^, define GVF as a vector field *V*(*x*, *y*)=(*u*(*x*, *y*), *v*(*x*, *y*)), and minimize energy generalization as follows:

(1) $$\begin{array}{c} F=\int \int u\left(u_{x}{}^{2}+u_{y}{}^{2}+v_{x}{}^{2}+x_{y}{}^{2}\right)+{\left|\nabla f\right|}^{2}{\left|V-\nabla f\right|}^{2}. \end{array}$$

According to the principle of variation, GVF satisfies Euler's equation

(2) $$\begin{array}{c} u\nabla^{2}u-\left(u-f_{x}\right)\left(f_{x}^{2}+f_{y}^{2}\right)=0. \end{array}$$

In the formula, *u* is a time-varying function, which changes continuously with time *t*, so we can get the following:

(3) $$\begin{array}{c} u\left(x,y,t\right)=u\nabla^{2}u\left(x,y,t\right)-\left(u\left(x,y,t\right)-f_{x}\left(x,y\right)\right)*\left(f_{x}{\left(x,y\right)}^{2}+f_{y}{\left(x,y\right)}^{2}\right),\\ \varpi =\max\sum_{i=1}^{n}\alpha_{i}-\frac{1}{2}\sum_{i=1}^{n}\alpha_{i}\alpha_{j}\beta_{i}\beta_{j}. \end{array}$$

### 2.2. Optic Canal Decompression

Visualization is a theory and a technique that can be used to convert data into graphics or images by displaying image processing techniques and computer graphics techniques [16–18]. The definition of “visualization” was first proposed by the National Science Foundation in the 1980s. After a series of measures, the “visualization of scientific computing” as a branch has been recognized worldwide. The main knowledge areas covered by this discipline include computer-aided design, computer graphics, computer vision, image processing, etc., which are very important technologies for dealing with issues such as decision analysis, data processing, and data representation. Because an optical model is necessary to explain the light of three-dimensional discrete data, the rational selection of optical models is an important factor in determining the rendering effect of neuroimaging data [19].

(4) $$\begin{array}{c} \frac{\Delta I}{I}=\left(\frac{\rho *E*\Delta s*\beta }{E}\right)=\rho *\Delta s*\beta . \end{array}$$

When Δ*s* approaching 0

(5) $$\begin{array}{c} \frac{\text{d}I}{\text{d}s}=-\left(\rho \left(s\right)*\beta *I\left(s\right)\right)=-\kappa \left(s\right)*I\left(s\right). \end{array}$$

As the conditions change, the image will also change with the discovery

(6) $$\begin{array}{c} I\left(s\right)=I_{0}\exp\left(-\int_{0}^{s}\kappa \left(t\right)\text{d}t\right),\\ t\left(s\right)=\exp\left(-\int_{0}^{s}\kappa \left(t\right)\text{d}t\right). \end{array}$$

From this, we can see the following:

(7) $$\begin{array}{c} \partial =1-t\left(s\right)=1-\exp\left(-\int_{0}^{s}\kappa \left(t\right)\text{d}t\right). \end{array}$$

When Δ*s* approaches zero, use the following differential equation to illustrate the change in light intensity:

(8) $$\begin{array}{c} \frac{\text{d}I}{\text{d}s}=T\left(s\right)*\rho \left(s\right)*A=T\left(s\right)*\kappa \left(s\right),\\ I\left(s\right)=I_{0}+\int_{0}^{s}g\left(t\right)\text{d}t. \end{array}$$

For the application of diagnostic imaging in medical treatment, we generally adopt the following formula:

(9) $$\begin{array}{c} x\left(k+1\right)=Ix\left(k\right)+Jv\left(k\right),\;k=1,2,\ldots . \end{array}$$

The quadratic performance indicators are as follows:

(10) $$\begin{array}{c} K=\sum_{k=1}^{\infty }\left[x^{i}\left(k\right)Jx\left(k\right)+r^{i}\left(k\right)cJ\right],\\ f\left(x\right)=\sum_{i}^{n}\alpha_{i}\beta_{i}+\exp\left(-\left(\frac{{\left\|x_{i}-x_{j}\right\|}^{2}}{2x^{2}}\right)\right). \end{array}$$

Before the emergence of visualization technology, medical staff can only use two-dimensional images as a basis for judgment, and there are three ways of observation: axial, sagittal, and coronal [20]. In this way, the doctor's judgment will inevitably be added, which will have a great impact on the accuracy of the diagnosis. With the development of science and technology, especially in the development of microcomputer technology, visualization technology is widely used and utilized, and it greatly contributes to the improvement of the diagnosis accuracy of the doctor. However, with the development of medicine, the requirements for visualization and computers are getting higher and higher. Therefore, computer-aided technology has emerged. Computer-aided technology is not limited to three-dimensional visualization technology. It also involves image processing technology and computer graphics technology and so on that are convenient. Through reconstruction, virtual endoscopy, and roaming, and other technologies, the two-dimensional image is converted into a three-dimensional figure, and then the part that the doctor wants to see is displayed according to the requirements. Improve the diagnosis and treatment of doctors with better and more comprehensive help, reduce the doctor's subjective judgment, and improve the accuracy of diagnosis [21].

At present, there is no software system specifically for visualizing optic canal decompression surgery at home and abroad. Doctors can only perform analysis based on a two-dimensional CT image or a regular image workstation and can make a decision based on their experience. They cannot provide more accurate and accurate analyses to doctors. Careful help, and because optic canal decompression surgery is highly dangerous, and the location of the optic canal varies from person to person, so far, few doctors at home and abroad can undertake such an operation [22]. In order to help doctors better solve the problem of optic canal decompression surgery, medical staff in my country rely on computer visualization technology, computer graphics technology, image processing technology, and medical-related imaging technology to segment the optic canal and internal carotid artery using image segmentation and reconstruction technology reconstructs the three-dimensional model of the optic canal and internal carotid artery and displays them together. The roaming technique then determines the operation path, and the core of the operation is connected to the navigation via the reverse DICOM. This helps doctors determine the relative position of the optic nerve and internal carotid arteries and the state that may be encountered during surgery. Significantly improve the safety, accuracy, and minimally invasiveness of surgery, and reduce the pain of patients [23, 24].

### 2.3. Postoperative Care

All patients were admitted to the neurosurgical intensive care unit for postoperative follow-up, and statistical analysis showed that sending the patient to the intensive neurosurgery intensive care unit could allow the patient to receive good treatment and improve prognosis. Provide patients with vital signs, neurological function assessment, continuous cardiopulmonary monitoring, vital signs, and other monitoring [25]. The posture can achieve different therapeutic effects or reduce the corresponding complications. You can reduce the side effects of the anesthetic when you lie down and lie down. 6 hours later, the high position of the head and lower the foot 15 degrees lower can be beneficial for intracranial venous regurgitation, reducing the oxygen consumption of the brain tissue and reducing pneumonia and aspiration pneumonia.

1. Management of restlessness and pain: severe restlessness and pain lead to an increase in the body's stress response. Pain is an important cause of delirium. These factors increase the burden of vital organs and affect the prognosis. Sedation therapy can prevent the increase in blood pressure and reduce rebleeding, and the protective effect of brain tissue has also been clinically recognized [26]. Patients with agitation are given midazolam or dexmedetomidine sedatives, and patients with pain are given analgesic pumps or dezocine analgesics to reduce the adverse irritation caused by pain.
2. Blood pressure management: the fluctuation of blood pressure is closely related to the expansion of hematoma and poor prognosis, so the management of postoperative blood pressure is particularly important. At present, the optimal decision for blood pressure management is still unclear, and there is no large study that can confirm that an exact blood pressure target value can benefit widely or that rapid blood pressure reduction is absolutely harmful; some exploratory studies have shown that excessive blood pressure variability indicates a poor prognosis and it is recommended to avoid excessive fluctuations in blood pressure as the goal of blood pressure management. It is recommended that the blood pressure does not drop too fast or too low.
3. Management of blood sugar: in neurosurgery, due to stress reaction, elevated blood glucose is common in patients. Hyperglycemia has a positive correlation with a head injury. Initial elevation of blood glucose is an index that reflects the severity of the head injury and suggests a poor prognosis. Hyperglycemia worsens brain edema simultaneously. Blood glucose damages the immune function of the body and increases the probability of infection. Therefore, hyperglycemia is associated with a poor prognosis and an increase in mortality. At present, the best management methods and target values for blood glucose in patients with cerebral hemorrhage are different, and it remains to be studied [27]. After the operation, the blood glucose monitor was used to monitor the 2 h postmeal and fasting blood glucose, and at the same time, adjust the blood glucose measurement interval and the blood glucose treatment plan according to the monitored blood glucose situation, and give the inverted sugar liquid input to those with elevated blood glucose to control the blood glucose intake; the appropriate unit of insulin and glucose is mixed in the vein according to the condition of the blood sugar level. To the patient who is taking gastrointestinal nutrition regularly, subcutaneous injection of a short time active insulin 15 minutes before the meal stabilizes the blood sugar level from 6 to 10 mmol/L.
4. Liquid management: fluid management is an important part of the management of critically ill patients, involving the resuscitation and maintenance of the patient's volume, as well as the control of intracranial pressure. After the operation, patients need to be given supplementary fluids and adequate nutrition for physiological needs [28]. In general, it is recommended to use an aqueous solution as a maintenance solution for primary choice in a neurosurgical patient, to compensate for the need for daily and excess moisture, and to compensate for the electrolyte to prevent electrolyte damage. Routinely give 2000–2500 ml fluid and decide whether to give 20% manna according to the specific situation. Dehydrating drugs such as alcohol reduce intracranial pressure. Insufficiency of nutrition can increase complications, and strengthening nutritional support can improve the prognosis of patients has become a consensus. For those who cannot eat by mouth, nasal feeding is given, and 20–25 kca/(kg·d) is used as the energy supply goal in the acute phase.
5. Body temperature management: elevated body temperature is a powerful vasodilator, which can increase intracranial pressure and increase brain metabolism rate, and may also lead to hematoma enlargement, which is extremely unfavorable for the prognosis of patients with cerebral hemorrhage. The duration of fever is also closely related to the prognosis. Actively search for the cause of fever and treat it. Physical cooling is a simple, effective, and safe way to cool down. Warm water baths, alcohol cooling, etc., are given, and an indomethacin suppository is given to the anus [29–31].
6. Imaging examination: CT should be reviewed as soon as possible after the operation, which can improve the accuracy of the calculation of hematoma clearance rate and reduce the error caused by postoperative bleeding; it also reduces the confusion caused by residual hematoma after hematoma or rebleeding. The CT reexamination time in this study was all after the patient's spontaneous breathing recovered and the reexamination immediately, no more than 24 hours after the operation.

Human cells have plasticity and functional reorganization. This is theoretical support for superior rehabilitation effects of neurological disorders that are recognized in the rehabilitation circle. Rehabilitation therapy occupies an important place in the treatment process, and the recovery time window has attracted people's attention. As a medical staff, in the process of preventive medication for patients, the patient's own economic situation should be fully considered. When the economic level permits, patients should be advised to take cost-effective and effective drugs as much as possible, and patients should be encouraged to take the drugs for a long time. Medication compliance shortens the distance between clinical practice and prevention guidelines.

## 3. Nursing Experiment of Optic Canal Decompression for Treatment of Traumatic Vision Disorders

### 3.1. Preoperative Preparation

Before the operation, fasting water, routine CT examination, CT scan with a thickness of 0.5 cm to obtain CT images, give ECG monitoring to monitor vital signs, continue to inhale oxygen, give nicardipine 5–15 mg/h continuous intravenous infusion to reduce blood pressure, if necessary, and give 20% mannitol dehydration to reduce intracranial pressure. Perform routine fasting and drinking before surgery, establishing intravenous access after entering the room, monitoring blood pressure, heart rate, breathing, pulse, and other vital signs, and administer dexmedetomidine, propofol, sufentanil, and other anesthetics.

### 3.2. Surgical Steps

(1) Make a small side nasal incision on the affected side first, and then cut the area from the inner end of the brow arch to the upper part of the alar, but do not cut the alar. (2) Open the nasal bone plate and enlarge the bone hole to ensure that the bone hole is in the area between the nasal root and the lacrimal sac. Then, use curettage to remove the ethmoid sinus anterior and posterior groups, and the scraping range is from the lamina to the upper jaw. The area between the upper boundary of the sinus will reach the anterior boundary of the sphenoid sinus after the above operations. (3) Remove the anterior inferior wall of the sphenoid sinus and open the sphenoid sinus cavity. If you encounter edema mucosa and blood clots, you can directly clear them. (4) After opening the sphenoid sinus, there will be a posterior obliquely upward skeletal protrusion called the optic canal. (5) Determine whether the optic nerve sheath needs to be cut according to whether there is edema in the optic canal. Generally, a scalpel is used to make a few tiny openings on the sheath to relieve pressure.

### 3.3. Data Sources

The data in this article are mainly obtained from the clinical data of the inpatient's diagnosis, the patient's understanding of the scene and the statistics of the telephone interview. The newly diagnosed patients with visual impairment in our hospital from November 2019 to March 2020 were selected. Then statistical data is categorized, analyzed, and simulated by computer software. We conduct investigations on doctors and patients, respectively, and conduct nursing work for the treatment of traumatic visual impairment by optic canal decompression under the intelligent Internet of Things medical nasal endoscopy. The evaluation method is based on the entropy method and comprehensive quantitative and qualitative analysis.

### 3.4. Statistics

All data analysis in this article uses SPSS19.0, and statistical test uses two-sided test, significance is defined as 0.05, and *P* < 0.05 is considered significant. The statistical results are displayed as mean ± standard deviation (*x* ± SD). When the test data obey the normal distribution, the double *T* test is used for comparison within the group, and the independent sample *T* test is used for comparison between the groups. If the regular distribution is not sufficient, two independent samples and two related samples will be used for inspection.

## 4. Analysis of Nursing Experiment of Optic Canal Decompression for Treatment of Traumatic Visual Disorder

### 4.1. Distribution of Patients

We have collected statistics on people who have undergone treatment for visual impairment in city hospitals, classified patients who have been treated for visual impairment in recent years, and classified patients according to the causes of visual impairment, as shown in Table 1.

From Figure 2, we can see that the number of visually impaired patients in our province showed a trend of rising first and then falling. It was at the peak of the number of patients in 2014 and 2015. However, with the continuous advancement of medical technology in recent years, the number of patients is increasing. It is classified according to factors such as age and gender of the population. I hope to find out the characteristics and rules of visual impairment. The specific data are shown in Table 2:

From Figure 3, we can see that among the patients admitted to the hospital, there are patients of all ages, but the age of the main patients is between 20 and 40 years old, reaching about 60%. This shows that when treating vision disorders, we must pay attention to the way of treatment and rehabilitation takes into account the acceptance level of patients in this age group in order to achieve better treatment results.

### 4.2. Differences in Imaging of Visual Impairment

We examine different patients and count the various parameters of the patients to check the severity of the visual impairment of the patients and divide them into four categories: congenital, benign, trauma, and internal trauma. The classification parameters are shown in Table 3.

As shown in Table 3, we use dynamic capture and static capture parameters to classify visually impaired patients into four categories: congenital, benign, trauma, and internal injury. From the table, we can clearly see that there are obvious differences in the parameters of different types of patients. The difference between benign and traumatic values is about 60. It is obvious from the chart that we display different types of visually impaired images, as shown in Figures 4–6.

### 4.3. Nursing Prognosis

We classify the patients with visual impairment, collect statistics on the patients' living habits and physical conditions, and obtain the causes of the patients' visual impairment, and then carry out targeted rehabilitation and prognosis so that the patients can recover. The details are shown in Tables 4 and 5.

From the table, we can see that bad living habits are an important reason for the difficulty in nursing and rehabilitation of patients. Most patients have the habit of smoking and drinking, which causes the patients' own high blood fat and high blood pressure to be more serious, which greatly hinders them. We compare the rehabilitation prognosis of patients with normal schedules and patients with bad habits, as shown in Figure 7.

From Figure 7, we can see that compared to patients with normal programs, patients with bad programs have much lower speed and efficiency of recovery, which shows that good living habits are extremely important for the prognostic recovery of patients. When rehabilitating visually impaired patients, we should pay attention to the patients' living habits in order to better recover the patients.

## 5. Conclusion

The internal carotid artery is close to the optic canal and is located in the cavity of the sphenoid sinus. The structure is complex. The method of realistically rebuilding the structure is the study task of this article. Since the internal carotid artery around the optic nerve has a C-shaped structure, it is difficult to obtain the structural image. It is relatively large, so this article adopts sampling based on the smart medical Internet of Things. All the structures of the internal carotid artery around the optic canal are presented on a two-dimensional image. The technology of mapping the two-dimensional space position to the three-dimensional space is a good realization of the operation. Connecting optic canal decompression surgery with smart medical care cannot only achieve surgical planning but also real-time observation, effectively reducing surgical risks. High technology promotes the rapid development of this medical device. 3D endoscopy has a three-dimensional effect. It has been invented and used in clinics and will gradually replace ordinary endoscopes. The combination of nasal endoscopy and intraoperative imaging technology will make the effect of endoscopic surgery more obvious. The combination with artificial intelligence in the future is also a development trend, and there may be more minimally invasive new surgical methods used in the clinic.

## Figures and Tables

**Figure 1:** The application of endoscopy in medicine (from image.baidu.com).

**Figure 2:** Number of visually impaired patients.

**Figure 3:** Age distribution of patients.

**Figure 4:** Schematic diagram of patient intranasal classification (from image.baidu.com).

**Figure 5:** Schematic diagram of intranasal classification of patients with internal injuries (from image.baidu.com).

**Figure 6:** Schematic diagram of intranasal classification of trauma patients (from image.baidu.com).

**Figure 7:** Rehabilitation effect of patients with different lifestyle habits.

**Table 1:** Causes of visual impairment in recent years.

Causes	2011	2012	2013	2014	2015	2016	2017	2018	2019	2020
Corneal scar	24	34	38	25	27	35	39	30	28	34
Corneal degeneration	29	24	26	34	33	29	37	41	46	43
Congenital visual impairment	21	17	16	13	22	9	11	15	10	21
Caused by trauma	24	25	29	31	25	29	33	35	37	40
Unknown reason	23	25	34	29	26	34	36	35	39	41

**Table 2:** Classification of people with visual impairment.

	Corneal scar	Corneal degeneration	Congenital visual	Caused by trauma	Unknown reason
0–12	3	8	11	7	8
13–26	66	88	31	47	18
27–45	57	61	99	36	26
46–60	32	91	87	53	13
Over 60	27	42	51	21	9

**Table 3:** Patient SPN classification.

	Congenital	Benign	Internal injury caused	Caused by trauma	*P*
Optic nerve	83.88 ± 3.77	78.56 ± 8.23	88.35 ± 5.78	79.26 ± 2.38	*P* < 0.05
Filter	5.69 ± 4.32	8.79 ± 3.58	17.23 ± 4.85	15.32 ± 3.51	*P* < 0.05
Daily life	12.34 ± 5.81	7.56 ± 4.25	8.48 ± 3.45	5.23 ± 2.01	*P* < 0.05
Motion capture	9.24 ± 3.52	13.52 ± 4.72	27.89 ± 5.32	25.34 ± 3.17	*P* < 0.05
Static capture	4.25 ± 2.35	9.25 ± 3.14	12.47 ± 4.91	11.37 ± 4.17	*P* < 0.05

**Table 4:** Living habits of patients.

Risk factors	Cardiogenic infarction	Noncardiac infarction	Sum	*P*
Age ≥75	35	21	56	0.038
Male	60	18	78	0.052
Smoking	34	9	43	0.032
Drinking	22	7	29	0.014
Hypertension	82	37	119	0.013
Diabetes	32	12	44	0.023
Hyperlipidemia	34	13	47	0.027
Hyperhomocysteinemia	46	24	70	0.095

**Table 5:** Living habits of patients.

Risk factors	OR	95% CI	*P*
Age ≥75	0.935	0.378–1.853	0.038
Male	1.325	0.628–2.987	0.052
Smoking	1.337	0.425–3.286	0.032
Drinking	2.014	0.537–7.638	0.014
Hypertension	0.382	0.172–1.253	0.013
Diabetes	1.079	0.489–2.356	0.023
Hyperlipidemia	3.158	1.289–7.895	0.027
Hyperhomocysteinemia	0.856	0.477–2.235	0.095

## Data Availability

No data were used to support this study.
